# Reliability and validity of a video-based markerless motion capture system in young healthy subjects

**DOI:** 10.1016/j.heliyon.2025.e42597

**Published:** 2025-02-12

**Authors:** Ziqi Wang, Hao Chen, Lei Yue, Jianming Zhang, Haolin Sun

**Affiliations:** a Department of Orthopedic, Peking University First Hospital, China; b Department of Rehabilitation Medicine, Peking University First Hospital, China

**Keywords:** Gait, Markerless motion capure system, Three-dimensional motion analysis system, Reliability, Validity

## Abstract

**Background:**

Gait analysis is widely utilized for the diagnosis and prognosis of various diseases. Recently, innovative convenient markerless motion capture systems have been developed to replace the traditional marker-based three-dimensional motion capture systems.

**Purpose:**

s:This study is to evaluate the test-retest reliability of a novel video-based markerless motion capture system(Watrix, China) and to assess its concordance with a three-dimensional motion analysis system (BTS, Italy) in a population of young healthy subjects.

**Participants and methods:**

Our study included 36 healthy adult participants. Each subject underwent three assessments using Watrix system and BTS system. To evaluate the validity and reliability of the measurements, we employed paired-sample t-tests, Wilcoxon signed-rank tests, intra-class correlation coefficients, Bland-Altman analysis and Passing Bablok regression analysis.

**Results:**

Both intra-rater and inter-rater reliability demonstrated moderate to excellent correlations, with intraclass correlation coefficient (ICC) values ranging from 0.507 to 0.936, except for cadence(ICC = 0.233). The validity exhibited a good correlation for sagittal plane parameters(ICC ranging from 0.818 to 0.883) and a moderate correlation for the coronal and transverse parameters (ICC ranging from 0.520 to 0.608). The Passing Bablok linear regression analysis indicated that the confidence intervals for the intercepts of all parameters included 0, while the confidence intervals for the slopes of most parameters encompassed 1 except for step width, pelvic obliquity, and hip adduction-abduction angle. The implementation of Watrix system significantly decreased the testing duration for participants.

**Conclusions:**

The Watrix system demonstrated relatively high test-retest reliability. The Watrix and BTS systems demonstrated moderate to good agreement for most parameters. However, the Watrix system tended to underestimate coronal and transverse plane parameters, resulting in lower consistency. In addition, the markerless motion capture system greatly reduces the testing duration.Optimizing algorithms to improve recognition accuracy remains the main direction of research.

## 1 Introduction

Gait refers to the posture and movement of an individual while walking, encompassing the intricate coordination of the body's muscles, tendons, soft tissues, bones, joints, and nerves. Deviations from the typical gait pattern are often indicative of specific neurological, muscular, or skeletal pathologies [1]. Consequently, gait analysis has been extensively utilized as a diagnostic and prognostic tool in various fields, including orthopedics [2], neurology [3], sports medicine [4], rehabilitation [5] and forensic medicine [6]. Accurately identifying gait-related parameters is essential for effective assessment and intervention. Traditional movement analysis typically depends on patient self-reports, practitioner observations, and visually assessed rating scales for disease diagnosis, monitoring, and treatment. However, these methods are inherently subjective and susceptible to errors due to variability in individual interpretation [7].

To accurately evaluate gait, 3D Motion Capture (MOCAP) is used, combining infrared cameras, reflective sensors, and force plates, making it the gold standard in quantitative gait analysis [8]. These systems provide quantitative and objective data regarding spatiotemporal parameters, electromyography, and ground reaction forces. Traditionally, motion capture (MOCAP) gait analysis has been conducted in controlled laboratory environments, necessitating large testing spaces and precise conditions, which limit its feasibility for clinical applications [9]. Moreover, the complexity and time required for data collection and processing, along with challenges such as soft tissue artifacts [10] and the inability of cameras to consistently track specific markers due to occlusions [11], further restrict the applicability of MOCAP systems in clinical and sports settings. Over the past decade, advancements in hardware development and artificial intelligence (AI) have facilitated the emergence of markerless motion capture (MMC), which integrates AI with high-speed video technology. This approach enables gait analysis in constrained and dynamic environments, offering a viable alternative to traditional laboratory-based motion capture systems.

The accuracy of 2D pose estimation models is well validated [12,13], but their single-frame basis limits motion parameters, requiring 3D markerless motion capture for precise gait analysis. The single-camera markerless system also demonstrated good agreement; however, it required a greater number of test trials and exhibited limitations such as reduced accuracy at image edges and the inability to provide multi-plane parameters [[14], [15], [16]]. Several studies have validated the effectiveness of 3D markerless gait analysis systems in measuring spatiotemporal and kinematic parameters [[17], [18], [19], [20]]. However, the supporting evidence remains limited [21,22], highlighting the need for further validation to ensure their reliability and accuracy [23].

This study aimed to compare two motion capture systems for quantitative gait analysis in healthy adults: a simple 3D MMC system (Watrix, China) using multiple depth cameras and a pose estimator, versus the gold standard MOCAP system (BTS, Italy). Our main hypothesis is that, compared to MOCAP, the markerless system will measure spatiotemporal parameters and the kinematic parameters with good accuracy in multiple planes. The secondary hypothesis suggests that markerless system will exhibit excellent test-retest reliability.

## 2 Materials and methods

### 2.1 Participants

According to Walter [24] et al., the sample size was determined based on a minimum acceptable Intraclass Correlation Coefficient (ICC) (p0) of 0.75 and an anticipated ICC (p1) of 0.90. This calculation indicated that a total of 36 subjects was necessary for the study. Ultimately, the sample consisted of 36 subjects.

The inclusion criteria for this study are as follows: participants must be aged between 18 and 40 years; they must not exhibit any symptoms, including but not limited to back pain, lower limb pain, numbness, or weakness; there should be no observable abnormalities in the bones and joints; participants must demonstrate normal active and passive range of motion, exhibit normal muscle tone, and present with no pathological signs; finally, participants should be able to walk smoothly without experiencing any discomfort during the walking process.

Exclusion Criteria: Individuals with a history of spinal, limb bone, or joint surgery and trauma; those with mental disorders, cognitive impairments, or other psychiatric conditions; patients with diseases that impact gait and walking distance, including but not limited to limb vascular disease, cerebral infarction, heart failure, Parkinson's disease, cerebellar disorders, and muscle weakness; as well as pregnant and lactating women.

Eventually, the study included a total of 36 participants, consisting of 20 males and 16 females, all of whom demonstrated normal gait patterns. Comprehensive details pertaining to the fundamental characteristics and physiological measurements of the participants are presented in Table 1. There were no instances of missing data.

**Table 1:** Baseline information.

N = 36 (male = 20,female = 16)	Mean ± SD	Min	Max
**Age(years)**	23.72 ± 3.28	20	33
**BMI(kg/m**^**2**^**)**	22.55 ± 3.83	16.41	33.41
**Weight(kg)**	65.58 ± 15.70	42	104
**Height(m)**	1.69 ± 0.09	1.5	1.82
**ASIS breadth(cm)**	26.42 ± 2.44	23	34
**Right pelvis depth(cm)**	9.49 ± 1.30	6	11.7
**Left pelvis depth(cm)**	9.55 ± 1.36	5.8	12.7
**Right leg length(cm)**	85.58 ± 5.81	76	95
**Left leg length(cm)**	85.94 ± 5.86	75	95
**Right knee diameter(cm)**	9.27 ± 0.97	7	11
**Left knee diameter(cm)**	9.16 ± 0.99	7	10.8
**Right malleolus diameter(cm)**	7.01 ± 0.87	5.5	9
**Left malleolus diameter(cm)**	7.02 ± 0.91	5.5	9

The data is presented as mean and standard deviation(SD).

Min,minimum value; Max,maximum value.

### 2.2 Ethical aspects

The present study has received ethical approval and has been registered under the identifier CHiCTR2300068787. Approval was granted by the Ethics Committee of Peking University First Hospital on February 16, 2023 (No. 2022-183-002). Written informed consent was obtained from all participants involved in this research.

### 2.3 Gait analysis

The research was carried out at the Rehabilitation Department of Peking University First Hospital from November 2022 to February 2023. Two different systems were compared for gait analysis in healthy adults: the BTS SMART DX-400 System (BTS Bioengineering Corp., Milan, Italy) and the Watrix System (Watrix.AI Corp, China)(Fig. 1).

**Fig. 1:** Flowchart of the gait analysis.

#### 2.3.1 BTS system

The BTS SMART DX-400 is an optoelectronic system made up of eight infrared cameras functioning at an acquisition frequency of 100 Hz, two force plates (BTS® P6000D), one synchronous camera (BTS® eVixta, with an acquisition frequency of 40 Hz), a set of surface electromyography equipment, twenty-two retro-reflective passive markers and a data station for the recording and processing of information. Firstly, the subjects underwent measurements of anthropometric parameters. Then according to the Davis protocol [25], 22 markers are attached to specific locations on the body surface.These regions included the acromion, the C7 spinous process, the anterior superior iliac spine, the midpoint of the posterior superior iliac spine line, the greater trochanter of the femur, the lateral femoral condyle, the fibular head, the lateral malleolus, the calcaneus, the lateral edge of the fifth metatarsal, the middle third of the thigh, and the middle third of the tibia(Fig. 2A). To minimize errors arising from anatomical misidentification, marker placement was jointly verified by two operators [26]. Subsequently, participants were allowed to ambulate freely within the laboratory for a duration of 5 min, thereby enabling them to acclimate to the environment.

**Fig. 2:** (A) Markers labelling of marker-based motion capture system (B) Markerless motion capture system identifing key points of the human body (C) Schematic diagram of key points in video recognition.

Participants were instructed to stand barefoot for a duration of 5 s to assess their static parameters. Following this, they were directed to walk along a designated pathway in a single direction to collect kinematic parameters. Two stable gait cycles were selected for data extraction. The BTS Smart Analyzer was employed for the analysis of these parameters, and average values were calculated for subsequent statistical analysis. This procedure was repeated three times to complete a single test, and the resulting data were averaged to enable a comprehensive gait analysis.

#### 2.3.2 Watrix system

The Watrix system utilized in this study is a markerless motion capture system developed by WATRIX AI Company (China). It consists of six high-definition cameras and a data processing server, which can ultimately output reports to devices such as mobile computers through the network. The markerless gait analysis system in this study utilizes a convolutional neural network (CNN)-based AI algorithm for automatic human keypoint localization. CNNs extract hierarchical spatial features from video frames, progressively learning human anatomical structures. The algorithm first generates heatmaps to estimate keypoint probability distributions, identifying joints such as the hip, knee, and ankle. A part affinity field (PAF) is then applied to link keypoints and reconstruct the skeletal structure. This approach enables accurate gait tracking without physical markers, making it suitable for natural, unconstrained environments(Fig. 2B and C). By integrating temporal information across consecutive frames, the system improves robustness against occlusions and viewpoint variations. The resulting joint trajectories and kinematic parameters provide a reliable foundation for gait assessment, supporting applications in clinical diagnostics, rehabilitation monitoring, and biomechanics research.

Upon arrival at the testing site, participants were instructed to walk freely for a duration of 5 min to acclimatize to the environment. Following this acclimatization period, participants stood in the designated recognition area for 5 s to record static parameters. Subsequently, they were directed to walk unidirectionally along the walkway to obtain kinematic parameters. Two stable gait cycles were selected for data extraction pertinent to gait analysis. This procedure was repeated three times to complete a single test, and the resulting data were averaged for the purpose of gait analysis. To verify the test-retest reliability of the system, each participant underwent a total of three tests. Operator A and Operator B completed one test on each subject on the same day. One week later, operator A conducted another test on the subjects.

### 2.4 Gait measurement

This study assessed the reliability of the Watrix system and conducted a comparative analysis with the BTS system across multiple dimensions, including spatiotemporal parameters, kinematic parameters, and assessment duration. The spatiotemporal parameters examined comprised step length, stride length, step width, cadence, and mean velocity. Kinematic parameters included sagittal plane measures such as the range of motion (ROM) of the hip, knee, and ankle joints, coronal plane parameters including hip adduction and abduction angles and pelvic tilt angle, as well as transverse plane parameters such as pelvic rotation angle. Furthermore, the time required for each system to complete the preliminary subject assessment was recorded.

### 2.5 Statistical analysis

The data are presented as means and standard deviations. Statistical processing and analysis were conducted using IBM SPSS Statistics version 25.0. Statistical significance was established at a threshold of P < 0.05. Intra-Class Correlation (ICC) and r values were interpreted according to the following criteria: excellent (>0.9), good (0.76–0.9), moderate (0.5–0.75), and poor (less than 0.50) [27]. The intra- and inter-rater reliability of Watrix system was assessed, along with the consistency between Watrix system and BTS system, utilizing Bland-Altman analysis. In this analysis, the mean score is plotted on the x-axis, while the mean difference is plotted on the y-axis. The width of the limits of agreement and the distance of the mean of the differences from zero serve as indicators for interpreting measurement errors. Bland-Altman plots facilitate comparisons among different measurement systems, observers, or sessions to evaluate the level of agreement [28]. Passing bablok linear regression is also used to analyze the consistency between Watrix system and BTS system. This statistical method was selected for its robustness in handling measurement errors, enabling a more precise evaluation of agreement between different measurement systems [29]. The mean values for both the left and right sides were utilized to ensure that individuals were treated as the unit of analysis rather than individual limbs [30]. For normally distributed data, paired samples t-tests were employed, whereas Wilcoxon signed-rank tests were applied for non-normally distributed data.

## 3 Results

The intra-rater reliability exhibited a moderate to excellent correlation for the temporal and spatial parameters (ICC ranging from 0.610 to 0.924) and a good to excellent correlation for the range of motion (ICC ranging from 0.884 to 0.936) for Operator A. Conversely, the inter-rater reliability demonstrated a moderate correlation for the temporal and spatial parameters (ICC ranging from 0.507 to 0.599, except for Cadence(ICC = 0.233)) and a good to excellent correlation for standing angles (ICC ranging from 0.828 to 0.910). These findings indicate no statistically significant difference between the data obtained by Operators A and B (Table 2).

**Table 2:** Intra- and Inter-rater reliability of the Watrix® parameters.

	operator A		operator B	Intra-Rater Reliability		Inter-Rater Reliability	
	test 1	test 2	test 3	ICC(%95CI)	P1^a^	ICC(%95CI)	P2^b^
**Step Length(m)**	0.66(0.06)	0.67(0.05)	0.65(0.06)	0.786 (0.580–0.891)	0.805	0.599 (0.214–0.796)	0.557
**Stride Length(m)**	1.37(0.13)	1.39(0.13)	1.40(0.14)	0.924 (0.851–0.961)	0.105	0.708 (0.426–0.851)	0.387
**Step Width(m)**	0.08(0.03)	0.08(0.02)	0.08(0.03)	0.863 (0.730–0.930)	0.927	0.790 (0.588–0.893)	0.208
**Cadence(steps/min)**	110.3(8.9)	113.0(11.8)	114.6(13.0)	0.610 (0.235–0.801)	0.260	0.233 (-0.505-0.609)	0.021∗
**Mean Velocity(m/s)**	1.27(0.19)	1.28(0.13)	1.24(0.30)	0.705 (0.422–0.850)	0.395	0.507 (0.032–0.748)	0.726
**Hip Flex-Extension(deg)**	40.32(4.36)	40.75(4.31)	41.02(3.72)	0.909 (0.822–0.954)	0.906	0.910 (0.823–0.954)	0.080
**Knee Flex-Extension(deg)**	61.37(4.11)	61.46(3.69)	61.83(3.29)	0.884 (0.773–0.941)	0.749	0.828 (0.662–0.912)	0.342
**Ankle Dors-Plantarflex(deg)**	33.13(4.54)	33.65(5.04)	33.32(4.65)	0.936 (0.874–0.967)	0.433	0.910 (0.824–0.954)	0.658

The data is presented as mean and standard deviation(SD).

ICC,Intraclass Correlation Coefficient; CI,Confidence Interval.

∗,p-value <0.05.

a the statistical significance of test 1 and test 2.

b the statistical significance of test 1 and test 3.

In the Bland–Altman plots, the limits of agreement for various gait parameters were determined as follows: step length (−0.10 to 0.09 m), stride length (−0.15 to 0.11 m), step width (−0.03 to 0.04 m), cadence (−23.6 to 20.3 steps per minute), mean velocity (−0.29 to 0.34 m/s), and the range of motion (ROM) for the hip (−4.89 to 4.79°), knee (−4.69 to 4.96°), and ankle (−4.86 to 4.24°) between operators A and B (Fig. 3). Additionally, the limits of agreement for operator A were recorded as follows: step length (−0.11 to 0.12 m), stride length (−0.27 to 0.22 m), step width (−0.04 to 0.05 m), cadence (−32.9 to 24.3 steps per minute), mean velocity (−0.53 to 0.59 m/s), and ROM for the hip (−5.27 to 3.87°), knee (−6.06 to 5.14°), and ankle (−5.36 to 4.97°) (Fig. 4).

**Fig. 3:** Bland-Altman plots comparing the results of different operators for various parameters: step length, stride length, step width, cadence, mean velocity, hip flex-extension angle, knee flex-extension angle, and ankle dorsiflexion-plantarflexion angle.

**Fig. 4:** Bland-Altman plots comparing results obtained by operator A for various parameters: step length, stride length, step width, cadence, mean velocity, hip flex-extension angle, knee flex-extension angle, and ankle dorsiflexion-plantarflexion angle.

The gait parameters, as assessed using Watrix system and BTS system, are presented in Table 3. Statistically significant differences were identified in the average comparison angles between the two measurement systems (p < 0.05). For spatiotemporal parameters, the mean differences between the two systems were recorded as 0.06 m for step length, 0.18 m for stride length, 0.04 m for step width, 4.4 steps/min for cadence, and 0.10 m/s for mean velocity. Regarding kinematic parameters, the average difference in joint range of motion between the two systems was approximately 1° (ranging from 0.17° to 1.34°). Statistical differences were observed in most parameters between the two systems, except for cadence, ankle flexion-extension angle, and pelvic rotation. The validity exhibited a good correlation for the lower limb ROM in sagittal plane (ICC ranging from 0.818 to 0.883) and a moderate correlation for the parameters of coronal and transverse planes (ICC ranging from 0.520 to 0.608).

**Table 3:** Validity of the Watrix® parameters.

	Parameters		Watrix® vs. BTS®		
	Watrix®	BTS®	MD	P-value	ICC(%95CI)
**Step length(m)**	0.66(0.06)	0.60(0.06)	0.06	<0.001∗	0.484 (-0.012-0.737)
**Stride length(m)**	1.37(0.13)	1.19(0.13)	0.18	<0.001∗	0.508 (0.034–0.749)
**Step width(m)**	0.08(0.03)	0.12(0.05)	0.04	<0.001∗	0.419 (-0.139-0.704)
**Cadence(step/min)**	110.8(11.9)	112.2(12.0)	1.4	0.474	0.714 (0.439–0.854)
**Mean velocity(m/s)**	1.24(0.19)	1.14(0.18)	0.10	0.005∗	0.664 (0.340–0.829)
**Hip Flex-Extension(deg)**	40.7(3.82)	39.4(4.50)	1.34	0.005∗	0.883 (0.771–0.941)
**Knee Flex-Extension(deg)**	61.6(3.40)	60.6(4.08)	1.00	0.050∗	0.818 (0.643–0.907)
**Ankle Dors-Plantarflex(deg)**	32.97(3.66)	32.64(3.41)	0.33	0.496	0.800 (0.607–0.898)
**Pelvis Obliquity (deg)**	1.77(0.60)	2.66(1.06)	0.88	<0.001∗	0.608 (0.232–0.800)
**Pelvis Rotation (deg)**	3.40(1.41)	3.57(1.36)	0.17	0.514	0.520 (0.058–0.755)
**Hip Ab-Adduction (deg)**	3.81(0.71)	4.53(0.94)	0.72	<0.001∗	0.543 (0.104–0.767)

This table shows the validity of the Watrix® in spatio-temporal and ROM parameters.

MD,mean difference.

∗,p-value <0.05.

The PB linear regression analysis indicated that the confidence intervals for the intercepts of all parameters included 0, while the confidence intervals for the slopes of most parameters encompassed 1. However, exceptions were observed for step width, pelvic obliquity, and hip adduction-abduction angle (Table 4).

**Table 4:** Testing time of Watrix® and BTS®.

	Testing time	Min	Max	P value
**Watrix®(min)**	17.75(3.61)	10	25	<0.001∗
**BTS®(min)**	33.97(4.63)	25	43	

The data is presented as mean and standard deviation(SD).

Min,minimum value; Max,maximum value.

∗,p-value <0.05.

The Bland–Altman plots illustrated the limits of agreement for step length, stride length, step width, cadence, and mean velocity, which ranged from −0.08 to −0.19 m, −0.12 to −0.47 m, −0.13 to −0.06 m, −36.2 to 31.0 steps/min, and −0.30 to 0.61 m/s, respectively. Most of the differences in lower limb ROM in sagittal plane and coronal parameters measured by the two systems are within 5°(Fig. 5, Fig. 6, Fig. 7).

**Fig. 5:** Passing Bablok linear regression and Bland–Altman plots comparing results between systems for step length, stride length, step width, cadence.

**Fig. 6:** Passing Bablok linear regression and Bland–Altman plots comparing results between systems for mean velocity, hip flex-extension angle, knee flex-extension angle, ankle dorsiflexion-plantarflexion angle.

**Fig. 7:** Passing Bablok linear regression and Bland–Altman plots comparing results between systems for pelvis obliquity, pelvis rotation and hip ab-adduction.

We also assessed the testing duration for each subject utilizing two systems. In the absence of marker placement, the Watrix system demonstrated a significantly shorter testing time in comparison to the BTS system (Table 5).

**Table 5:** Passing-Bablok linear regression analysis.

	Slope	LB	UB	Intercept	LB	UB	RSD
**Step Length(m)**	1.24	0.77	2.00	−0.08	−0.55	0.20	7.37 %
**Stride Length(m)**	1.00	0.60	1.64	0.17	−0.62	0.66	7.93 %
**Step Width(m)**	0.50	0.20	0.86	0.03	−0.01	0.06	30.23 %
**Cadence(steps/min)**	1.30	0.88	1.96	−32.14	−104.5	12.15	7.69 %
**Mean Velocity(m/s)**	1.10	0.73	1.65	−0.03	−0.65	0.38	10.76 %
**Hip Flex-Extension(deg)**	0.87	0.72	1.08	6.96	−1.55	12.61	4.71 %
**Knee Flex-Extension(deg)**	0.84	0.59	1.13	10.75	−7.62	25.56	3.30 %
**Ankle Dors-Plantarflex(deg)**	1.17	0.78	1.64	−4.93	−20.31	7.41	6.26 %
**Pelvis Obliquity (deg)**	0.48	0.28	0.73	0.55	−0.13	0.94	28.65 %
**Pelvis Rotation(deg)**	1.24	0.69	1.78	−0.91	−2.92	0.88	33.20 %
**Hip Ab-Adduction (deg)**	0.61	0.35	0.93	1.14	−0.48	2.13	16.32 %

LB = Lower Bound of confidence interval; UB = Upper Bound of confidence interval.

RSD = Residual Standard Deviation.

## 4 Discussion

This study aims to compare the performance of the Watrix markerless motion capture system and the BTS SMART DX system in assessing the spatiotemporal and kinematic parameters of gait in healthy adults. Both intra-rater and inter-rater reliability demonstrated moderate to excellent correlations, with intraclass correlation coefficient (ICC) values ranging from 0.507 to 0.936, except for cadence (ICC = 0.233). Given that only cadence exhibited poor reliability, it is hypothesized that the Hawthorne Effect may have influenced the results. Participants, upon perceiving they were being observed, may have exhibited unstable gait behavior during testing, leading to measurement errors [44].The Bland Altman plot shows that all spatiotemporal parameters exhibit good consistency. In terms of range of motion, the average differences for both intra- and inter-rater are within 1°, and most differences are within ±5°, which is considered acceptable in clinical practice [31].

In relation to the Bland-Altman plot assessing the validity of the Watrix device, the proportions of data points falling outside the 95 % limits of agreement are as follows: 2 out of 36 for step length, 3 out of 36 for stride length, 2 out of 36 for step width, 2 out of 36 for cadence, and 3 out of 36 for mean velocity. Although statistical differences were identified between the Watrix system and BTS system, as indicated by the poor to moderate Intraclass Correlation Coefficients (ICCs) ranging from 0.419 to 0.705, a certain degree of consistency is observable in the Bland-Altman plot. This consistency suggests the potential applicability of the Watrix device. We also found a significant correlation between the range of motion of the hip, knee, and ankle joints measured by Watrix system and BTS system in the sagittal plane, the indicators in the coronal and transverse planes demonstrated only moderate consistency [32,33]. The Passing-Bablok linear regression analysis indicated that the 95 % confidence intervals (CIs) for the slopes of step length, stride length, mean velocity, and hip/knee/ankle flexion-extension encompassed 1, demonstrating good agreement between the Watrix system and the BTS system, with no evidence of proportional bias. However, the slopes for step width, pelvis obliquity, and hip abduction-adduction were significantly lower than 1, suggesting that the markerless system underestimated these parameters, indicating the presence of proportional bias. The 95 % CIs for the intercepts of all parameters included 0, implying that systematic bias between the two systems was not significant. Additionally, the RSD values for step width (30.23 %), pelvis obliquity (28.65 %), and pelvis rotation (33.20 %) were relatively high, indicating greater measurement variability in the markerless system for these parameters. We hypothesize that this discrepancy may be attributed to the number and positioning of cameras [34]. Therefore, further research is warranted to investigate optimal camera configurations.

Our research has several limitations: Firstly, due to site limitations, we were unable to place the video gait analysis system and the 3D gait analysis system in the same site, and therefore were unable to measure both systems simultaneously, which may be the main source of error [35]. Therefore, Passing-Bablok linear regression analysis was employed as a supplementary method, as it accounts for measurement errors and is particularly suitable for comparing the two systems in this study. Secondly, considering privacy concerns, participants were required to wear tight-fitting clothing and maintain consistent attire across both system tests. However, clothing may affect the AI-based recognition of human keypoints in the markerless system and contribute to soft tissue artifacts in the BTS system, potentially introducing measurement errors [36]. Besides, a total of 36 participants were included based on the calculated sample size; however, the results indicate that the sample size remains insufficient [37]. Future research will aim to expand the sample size and incorporate a more diverse population [38] to enhance the generalizability of the findings.

In addition to our study, numerous other investigations have reported similar findings. Tishya [39] et al. observed that the kinematic patterns exhibited similarities between the marker-based and markerless systems. However, in certain instances, the markerless system demonstrated increased trial-to-trial variability, exhibited a more pronounced knee varus "bump" during the swing phase, or failed to accurately track the subject. Robert [40] et al. conducted a study involving thirty healthy adult participants who walked on a treadmill while data were simultaneously recorded using eight video cameras and seven infrared optical motion capture cameras. This setup provided synchronized markerless and marker-based data for comparative analysis. The results indicated a root mean square deviation (RMSD) of less than 5.5° for all segment angles, with the exception of those representing rotations about the long axis of the segment. Jincong [41] et al. recruited 18 typically developing (TD) children and 10 children with developmental dysplasia of the hip (DDH) to compare the consistency between video-based gait systems and three-dimensional gait systems. The findings suggested that the intraclass correlation coefficients (ICCs) were generally high (ICC >0.7), indicating moderate to good relative reliability, and the Bland-Altman plot analysis revealed no significant systematic errors. Although these studies report the enormous potential of video gait analysis systems, their reliability evidence is still insufficient and needs further validation and improvement.

In recent years, an increasing number of innovative devices for gait analysis have been developed, yet each type of device has its inherent limitations. For instance, the video-based unlabeled gait analysis device utilized in this study is prone to errors arising from occlusions and variations in video quality. To address these challenges, integrating multiple types of devices for gait analysis presents a promising research direction. Among emerging methods, radar-based gait analysis, including technologies such as millimeter-wave radar and ultra-wideband radar, offers unique advantages [42]. Radar systems are cost-effective, portable, and capable of penetrating certain obstacles, making them a suitable complement to video-based analysis. The combined use of radar and video-based systems has the potential to mitigate the limitations of unlabeled gait analysis, providing a robust solution with significant prospects for future applications.

## 5 Conclusions

This study proposed a comparison between the markerless motion capture system(Watrix system), and the marker-based motion capture system(BTS SMART DX), for assessing gait-related parameters in healthy adults. The Watrix system demonstrated relatively high test-retest reliability. The Watrix and BTS systems demonstrated moderate to good agreement for most parameters. However, the Watrix system tended to underestimate coronal and transverse plane parameters, resulting in lower consistency. In addition, the markerless motion capture system greatly reduces the testing duration.Optimizing algorithms to improve recognition accuracy remains the main direction of research.

## Funding statement

This research was supported by the 10.13039/501100001809National Natural Science Foundation of China (No. 62471010).

## CRediT authorship contribution statement

**Ziqi Wang:** Writing – original draft, Visualization, Validation, Software, Resources, Methodology, Investigation, Formal analysis, Data curation, Conceptualization. **Hao Chen:** Resources, Project administration, Methodology, Investigation. **Lei Yue:** Formal analysis, Data curation. **Jianming Zhang:** Investigation. **Haolin Sun:** Writing – review & editing, Supervision, Conceptualization.

## Declaration of competing interest

All authors disclosed no relevant relationships.
